# A Multitask Deep Learning Framework for DNER

**DOI:** 10.1155/2022/3321296

**Published:** 2022-04-16

**Authors:** Ran Jin, Tengda Hou, Tongrui Yu, Min Luo, Haoliang Hu

**Affiliations:** ^1^College of Big Data and Software Engineering, Zhejiang Wanli University, No. 8 South Qianhu Road, Ningbo, China; ^2^Ningbo University of Finance & Economics, No. 899 College Road, Ningbo, China

## Abstract

Over the years, the explosive growth of drug-related text information has resulted in heavy loads of work for manual data processing. However, the domain knowledge hidden is believed to be crucial to biomedical research and applications. In this article, the multi-DTR model that can accurately recognize drug-specific name by joint modeling of DNER and DNEN was proposed. Character features were extracted by CNN out of the input text, and the context-sensitive word vectors were obtained using ELMo. Next, the pretrained biomedical words were embedded into BiLSTM-CRF and the output labels were interacted to update the task parameters until DNER and DNEN would support each other. The proposed method was found with better performance on the DDI2011 and DDI2013 datasets.

## 1. Introduction 

With the rapid development of biomedicine and the exponential growth of publications have made it hard to extract a number of drug-related information. It is essential to extract valuable information if we want to make the best of medical text. Medicine is a class of chemical substances that are highly associated with biological research. It is of vital significance to observe how to accurately capture the entity information as contained in medicine. Drug refers to chemical name, generic term, or brand name. As a chemical product usually has a complex name, the brand name may not exactly identify a drug in the expiry of relevant patents. For example, the drug “quetiapine” is associated with the brand name “Seroquel XR.” Therefore, a special generic term, which needs to be explicitly defined for drug approval, should be designed for standard scientific reports and labels. Drug-specific names are subject to tight control by WHO (World Health Organization) and some organizations in the USA and elsewhere. For example, the European Medicines Agency (EMA) finalized the naming scheme fit to drug function for ease of pronunciation and translation and developed some criteria that differentiate a drug name from others so as to avoid any transcription and replication error in the R&D process [1]. This would justify the automatic extraction of potential medical information from massive biomedicine-related publications as a crucial part of biomedical research and industrial medicine manufacturing.

Drug-Named Entity Recognition (DNER), which is intended to identify the drugs referred to in unstructured drug texts, is an underlying task of recognizing the span and type of the named entity subordinated to predefined semantic types. Unlike ordinary NERs (Named Entity Recognition), DNER generally consists of long label sequences and contains plenty of alternate spellings of synonyms and entities, resulting in the inefficiency of drug dictionary and hard detection of entity boundaries. In this regard, Drug-Named Entity Normalization (DNEN) is also believed to be a crucial task.

DNEN, which is intended to map the acquired DNERs to a controlled vocabulary, is usually considered a task subsequent to DNER. Both DNEN and DNER can be deemed as sequence labeling problems.  Figure 1 illustrates an example with respect to DNER and DNEN tasks, the input text contains the drug-specific name “Omeprazole” and the R&D organization “Astra Pharmaceuticals”, and the label of each word in the text and its entity ID are output.

As the naming scheme, evaluation criteria and cross-border synchronization have been developing dynamically for many years, and there is no definitive dictionary or grammar applicable to drug names; DNER and DNEN processes are subject to many challenges: (1) the rapid updates of drug-related knowledge make it hard for a handmade dictionary to meet actual needs; (2) language tends to be complex and there is a scarcity of high-quality label texts; (3) the simple modeling of DNER and DNEN cannot allow both processes to support each other.

It is intended that the proposed model can capture more resourceful semantic features and identify the representation of polysemous and ambiguous words in drug sequence, thus accurately recognizing drug names. A multitask deep learning model multi-DTR (Multi-Drug Tip Recognition) was proposed, and the principal contributions of this work were that text information can be exploited by extracting the character-level representations of words, embedding words based on biomedicine pretraining, and extracting the features by context-sensitive word embedding after ELMo (Embeddings from Language Models) training. To make the best of the training data, a multitask learning strategy was taken, which allows for the explicit feedback of DNER and DNEN and makes different tasks support each other.

This article is structured as follows: in Section 2, some related works on DNER and DNEN were presented; in Section 3, the proposed neural network framework was described; in Section 4, relevant datasets and parameter setups were briefed; in Section 5, the result of the assessment was reported in particulars; in Section 3, a conclusion was drawn.

## 2. Related Works

NER is one of the underlying tasks in NLP, but there are a limited number of related works on DNER [2–4]. The access to some large-scale biomedical corpora [5–7] has enabled some generic NER models to be widely used in DNER. Common methods applicable to DNER can be roughly categorized into rule-based methods [8], dictionary-based methods [9], and machine learning-based methods [10]. In the case of rule-based methods, a number of labor resources are required to lay down rules, but the ambiguity and variability of terms are overlooked. If the target text appears to be complex, rule-based methods are found with a low recognition rate [11]. Tsuruoka et al. [12] made use of logistic regression to learn string similarity measures from the dictionary and performed soft character matching to avoid large difference of association due to exact string matching. Hettne et al. [13] developed a rule-based method for term filtering and disambiguation, then merged dictionaries to recognize small molecules and drugs as contained in the text. Eriksson et al. [14] created a Danish dictionary to recognize Adverse Drug Event (ADE) that may potentially occur in unstructured clinical narrative text. Despite this, the actual application needs can hardly be met due to a lack of dictionary and rapid update of biomedicine terms. The machine learning-based NER is currently a prevailing research interest. Cocos et al. [15] used ZRNN coupled with pretrained word embedding to recognize ADE on Twitter. Zeng et al. [16] performed automatic searching of words and character-level features in drug texts on LSTM-CRF (Long Short-Term Memory-Conditional Random Field) structure. To date, BERT (Bidirectional Encoder Representations from Transformers) [17] is the great hit model in the sector of Natural Language Processing (NLP). In the case of BERT, a transformer encoder was used and the upper and lower layers of the model are fully connected by a self-attention mechanism so that text information can be better processed. Lee et al. [18] ran a large-scale pretraining in respect of BERT (treated as a basic model) on PubMed and PMC and then developed the BioBERT (Biomedical Bidirectional Encoder Representations from Transformers) model. Despite the extraordinary properties, this model caused an enormous consumption of hardware resources in the training process.

DNEN, also a key part of information extraction, is generally listed as a subtask [19, 20] for some biomedicine-related NLP assessment tasks. Kang et al. [21] normalized disease-specific names by constructing a symptom text model and performing a comparative analysis. Lee et al. [22] used a dictionary to look up and standardize the entity. Lou et al. [23] proposed a transition-based model applicable to the recognition and normalization of joint disease entity, but such model heavily relies on handmade features and task types.

## 3. Neural Network Framework

In this article, the character feature representations (e.g., amidopyrine, aminophenazone, and aminopyrine) of an input word were extracted through Convolutional Neural Networks (CNN). Next, the extracted character features and words were embedded and input to BiLSTM (Bidirectional Long Short-Term Memory). The two-way LSTM (Long Short-Term Memory) was used to capture two separate hidden states (forward and backward) of each sequence, obtain the context-sensitive information, then connect two hidden states until the final output is generated. In the final step, the output vector of BiLSTM was backfed to CRF for jointly modeling the label sequence. DNER and DNEN can give back to each other by the output of two tasks, reduce the load of calculations, and realize the enhancement effect of both tasks.

### 3.1. Embedded Layer

For deep mining of drug-related information in the input text, the features were extracted by pretrained word embedding, context-sensitive word embedding, and character embedding.

#### 3.1.1. Pretrained Word Embedding

The rapid development of deep learning technology has led to an extensive use of word embedding, which offers an alternative to numerical representation of text (such as Word2Vec [24] and Glove [25]). Yu et al. [26] found that embedding pretrained words into unlabeled data would have many NLP tasks significantly improved. As inspired by Glove [25], we used the word representation method based on global word frequency statistics to pretrain data on PMC (PubMed Central) and PubMed biomedical corpora and to embed pretrained word vectors into the model.

#### 3.1.2. Character Representation

Evidence has shown that character information is crucial for sequence labeling tasks [16, 27]. Colobert et al. [28] suggested that the integrity of words can be used to label words, and local features extracted by CNN are exploited to construct all feature vectors. Ling et al. [29] tried to use character-level two-way LSTM for POS labeling, but the result of the experiment indicates that the performance of character-level two-way LSTM highly resembles CNN, but a heavier load of calculations is requested. Santos et al. [30] was the first researcher who suggested using CNN to learn character-level representations of words and associate them with the representations of common words. A number of subsequent works [31, 32] supported that the word-level information (such as prefixes and suffixes) can be leveraged to the extent possible by character-based word representation. Zhao et al. [33] exploited attention-based CNN to capture the association between context-sensitive information and discontinuous words. Strubell et al. [34] proposed ID-CNN (Iterated Dilated Convolutional Neural Network) as the generally dilated CNN architecture that improves the computational efficiency to the extent possible. Chiu et al. [35] used CNN to extract character vectors of a specific length from the word-specific characters, cascade them with the encoded features, then transmit them through the convolutional layer and the max layer.

In this article, CNN was used to acquire the character-level representation of a word. As is seen from Figure 2, the feature encoding process as a part in Chiu et al. [35] was deleted, the Dropout layer was added to prevent overfitting of CNN, and we finally had a word-specific character vector.

#### 3.1.3. Context-Sensitive Word Embedding

ELMo, a language model based on features, can model words given the context. Unlike Word2Vec and other word sectors that use a simple lookup table to obtain the unique representation, the word sector in ELMo represents the function of the internal network state. Even for the same word, the word sector shows changes dynamically. Thus, it first adopts two-way LSTM for pretraining and the two-way concept of ELMo is reflected through the network structure, which comprises the forward LSTM model and the backward LSTM model. The construction of the model is shown in Figure 3.

ELMo comes with a task attribute and is a linear combination represented by the middle layer of biLM. With respect to a given word, biLM of a *L* layer can obtain the representation of 2*L* + 1:

(1) $$\begin{array}{c} ELMo_{k}=\sum_{j=0}^{L}wh_{k,j}^{LM},\\ R_{k}=\left\{x_{k}^{LM},{\overset{⟶}{h}}_{k,j}^{LM},{\overset{\leftarrow }{h}}_{k,j}^{LM}|j=1,\ldots ,L\right\}=\left\{h_{k,j}^{LM}|j=0,\ldots ,L\right\}, \end{array}$$

where *w* is the weight of softmax-normalized, *x*_*k*_^*LM*^ denotes the input initial word vector, ${\overset{⟶}{h}}_{k,j}^{LM}$ denotes the forward LSTM output, and ${\overset{\leftarrow }{h}}_{k,j}^{LM}$ denotes the backward LSTM output. The context-sensitive dynamic word embedding as obtained from the above can more accurately reflect the complex semantic and grammatical features of the text.

### 3.2. Sequence Labeling

Some deficiencies of the character-level model include the multiple growth of the effective sequence size and a lack of inherent meaning in the characters. Thus, RNN can be used to process time series data of any length using neurons with self-feedback. However, it was reported [36] that RNN is usually inclined to the nearest input of the sequence in practice and cannot process long-term dependencies. Certain variants based on recurrent neural networks, such as Gated Recurrent Unit (GRU) and LSTM, have proven extraordinary performance. Yang et al. [37] used GRUs at the character- and word-level to encode morphological and context-sensitive information. Huang et al. [38] were the first researchers who used BiLSTM for sequence sorting and results showed that this model is less dependent on word embedding and can capture two hidden states (forward and backward) of each sequence well with strong robustness.

Both DNER and DNEN can be seen as sequence labeling tasks. In this work, BiLSTM was used to model the input character-level information, pretrained word embedding, and contextualized word embedding. It inputs a vector sequence containing *n* words (*x*_1_, *x*_2_,…, *x*_*n*_), then calculates the hidden state sequence (*h*_1_, *h*_2_,…, *h*_*n*_), and outputs the label (*o*_1_, *o*_2_ ,…, *o*_*n*_). Finally, the equation with respect to an update of the LSTM unit would be as follows:

(2) $$\begin{array}{c} i_{t}=\sigma \left(W_{xi}x_{t}+W_{hi}h_{t-1}+W_{ci}c_{t-1}+b_{i}\right),\\ c_{t}=\left(1-i_{t}\right)*c_{t-1}+i_{t}*\;\tanh\left(W_{xc}x_{t}+W_{hc}h_{t-1}+b_{c}\right),\\ o_{t}=\sigma \left(W_{xo}x_{t}+W_{ho}h_{t-1}+W_{co}c_{t}+b_{o}\right),\\ h_{t}=o_{t}*\;\tanh\left(c_{t}\right), \end{array}$$

where *σ* is elementwise sigmoid function, *∗* is elementwise product, *x*_*t*_ denotes the input vector at *t*, *h*_*t*_ is the hidden vector (also referred to as “output vector”), it denotes the value of the memory gate, *c*_*t*_ denotes the cell state, *o*_*t*_ denotes the value of the output gate, *W*_*xi*_, *W*_*xc*_, and *W*_*xo*_ denote the weight matrix of different gates of the input *x*_*i*_, *W*_*hi*_, *W*_*hc*_, and *W*_*ho*_ are the weight matrix of the hidden state *h*_*t*_, and *b*_*i*_, *b*_*c*_, and *b*_*o*_ denote the offset vector. Then the final output vector $h_{t}=\left[{\overset{⟶}{h}}_{t},{\overset{\leftarrow }{h}}_{t}\right]$ can be obtained.

After the training of BiLSTM, the entity labeling of unlabeled words can be predicted from the output ht. But in DNER task, some impossible combinations may also exist in the predicted data. For example, the label “I-BRAND” must not immediately follow the label “B-DRUG” logically, which means that we have to consider the label information of neighboring data. CRF is an undirected graphical model that focuses on the sentence level, instead of each position. Therefore, some impossible combinations should be ruled out.

With respect to the input sequence *Y* = {*y*^1^, *y*^2^,…, *y*^*n*^}, *y*^*n*^ denotes the *i*th word vector of input, *Z* = {*z*^1^, *z*^2^,…, *z*^*n*^} is the label sequence of the input sequence *Y*, and *P* is the score matrix of output by BiLSTM, where *k* denotes score of the *j*th label of the *i*th word, and its score can be defined as follows:

(3) $$\begin{array}{c} s\left(Y,Z\right)=\sum_{i=0}^{n}A_{z_{i},z_{i+1}}+\sum_{i=1}^{n}P_{i,z_{i+1}}, \end{array}$$

where *A* is the transition score matrix, *A*_*i*, *j*_ denotes the conversion score from the label *i* to the label *j*, and *y*_0_ to *y*_*n*_ is the start and end label of a sentence. They are added to a set of possible labels. Thus, *A* is a matrix whose size is *k* + 2.

The loss function of CRF is composed of the actual path score and the total score of all possible paths; both scores are given as follows:

(4) $$\begin{array}{c} P_{\text{Realpath}}=e^{s\left(Y,Z\right)},\\ P_{\text{total}}=\sum_{\tilde{z}\in Z_{Y}}e^{s\left(Y,\tilde{z}\right)}, \end{array}$$

where *e*^*s*(*Y*, *Z*)^ denotes the score of the possible path along, where the *Z* label is generated on the word *Y* and *e* is a numeric constant. In the training course, the log probability of the correct label sequence is maximized.

(5) $$\begin{array}{c} \log\left(P\left(Z|Y\right)\right)=\log\left(\frac{P_{\text{Realpath}}}{P_{\text{total}}}\right),\\ \text{Lossfounction}=-\log\left(P\left(Z|Y\right)\right),=\left(\sum_{i=1}^{L}x_{iy_{i}}+\sum_{i=1}^{L-1}t_{y_{i}y_{i+!}}-\log\left(\sum_{\tilde{z}\in Z_{Y}}e^{s\left(Y,\tilde{z}\right)}\right)\right). \end{array}$$

The loss function of CRF is computed by formula (5), where *x*_*iy*_*i*__ denotes the emission score with the word index as *i* and the label index as *y*_*i*_ and *t*_*y*_*i*_*y*_*i*+1__ denotes the transmit score with the word index as *y*_*i*_ and the label index as *y*_*i* + 1_. Then, we can search for the optimal path using the Markov hypothesis, coupled with the Viterbi algorithm.

### 3.3. Multitask Learning Strategy

Multitask Learning (MTL) is a kind of joint learning through which the differences and connections between tasks can be effectively analyzed and modeled. Hard sharing, soft sharing, and hierarchical sharing are currently the most-used structures by MLT. Hard sharing stacks a given task on top of the sharing layer [39]. Soft sharing supports each task with separate models and parameters, and the internal information contained in each model can be accessed [40], but it may also lead to the inefficiency of parameters. Hierarchical sharing puts different tasks in different network layers [41], but it relies on the handmade hierarchical shared structure. For DNER, since the same entity has a number of synonyms and various forms of representations, exact matching or fuzzy matching as lookup methods of the dictionary may cause great challenges to detecting entity boundaries. However, this can be avoided by adding the DNEN task. Specifically, the output of DNER such as “B-DRUG” is an explicit signal indicating the start of drug entity so that the search space of DNEN can be reduced, vice versa. Therefore, two explicit feedback strategies were incorporated as a part of the multitask learning framework to simulate the reciprocal enhancement effect among different tasks.

A multitask learning framework resembling that proposed by Zhao [42] was used to enable DNER and DNEN to support each other and to enhance the generalization ability of the model. In the first step, the training set was divided into subsets applicable to *T* tasks: *D*_1_,…, *D*_*T*_ prior to the training process. In the training process, a training set *t* was chosen and the instance for random training (*w*_1:*n*_, *y*_1:*n*_^*t*^) ∈ *D*_*t*_ was acquired, where *w*_*i*_ ∈ *W* and *W* denotes the input set; *y*_*i*_^*t*^ ∈ *L*^*t*^ and *L*^*t*^ denotes the label set. The label specific to the task *t* was used to predict the label *y*_*i*_^*t*^ and update the label *y*_*i*_^*t*^ and then the updated parameters were backfed to the model for asynchronous training of DNER and DNEN, with the particular equation written as shown in Figure 4.where DNER(*w*_1_:*n*, *i*) and DNEN(*w*_1_:*n*, *i*) denote the DNER and the DNE normalized function with the word sequence *w*_1_, *w*_2_,…, *w*_*n*_ and the index *i* as inputs, *y*_DNER_^*i*^ is the output of entity recognition applicable to the named entity label, *y*_DNEN_^*i*^ is the output of the entity normalized function applicable to the entity vocabulary label, *v*_*i*_^DNER^ is the input of DNER multiclass classification function that denotes the input of BiLSTM-CNN and the explicit feedback of DNEN, *v*_*i*_^DNEN^ is the input of DNEN multiclass classification function that denotes the input of BiLSTM-CNN and the explicit feedback of DNEN. *U* is the matrix mapping from DNEN to DNER, and *V* is the matrix mapping from DNER to DNEN.


(6) $$\begin{array}{c} \text{DNER}\left(w_{1:n},i\right)=y_{\text{DNER}}^{i}=\arg\max y_{\text{DNER}}^{i}=f_{\text{DNER}}\left(v_{i}^{\text{DNER}}\right),\\ \text{DNEN}\left(w_{1:n},i\right)=y_{\text{DNEN}}^{i}=\arg\max y_{\text{DNEN}}^{i}=f_{\text{DNEN}}\left(v_{i}^{\text{DNEN}}\right),\\ v_{i}^{\text{DNER}}=v^{k}\circ \left(v^{k}+y_{\text{DNEN}}^{i}U\right),\\ v_{i}^{\text{DNEN}}=v^{k}\circ \left(v^{k}+y_{\text{DNER}}^{i}U\right),\\ F_{\theta }^{k}\left(x_{1:n},i\right)=v_{i}^{k}=h_{L,i}^{k}\circ h_{R,i}^{k}. \end{array}$$

In this article, a fully shared mode was adopted to make the BiLSTM-CNN layer shared among tasks, which means that all parameters as contained in the model would be shared, except for the output layer applicable to DNER and DNEN. This construction enables the proposed model to capture feature representations of different tasks and interactively give feedback to generate prediction sequences.

## 4. Network Training

In this section, we provided particular information in relation to raining neural networks, including corpus, hyperparameter, optimizer, and assessment criteria. PyTorch was used to deploy the model and run the proposed model on Nvidia GTX 1080.

### 4.1. Datasets and Preprocessing

Obtain data from the DDI2011 and DDI2013 challenge corpora to construct the data set for training the deep learning model, and preprocess the data set for training the deep learning model in the following ways: randomly divide the dataset into *T* subsets, and *T* is an integer greater than or equal to 2. Establish four alphabets of word, character char, label label, and feature for each subset. Each alphabet is a dictionary for storing {key: instance, value: index}, where key represents the stored key, value represents the stored value, instance refers to the word, and index refers to the index. Based on the four alphabets of each subset, two lists are established for each subset. The two lists contain four columns of data, respectively. The four columns of data in the first list are [words, chars, labels, features], and the four columns of data in the second list are [words_Ids, chars_Ids, labels_Ids, features_Ids].

In the experiment, the DDI2011 Challenge Corpus from the drug-medicine interaction task was used. The minidom module as a part of python was used to extract <sentence> and <entity> elements, get the essential test and entity information, create a list, and match and annotate the entity and text. Next, all training datasets were collected as training data, and all test datasets were collected as test data. In this work, the sample was preprocessed using BIO labeling, where B denotes the first token of the entities in the sample, I denotes the token in the entity, and *O* denotes the token that does not fall into the category of entities.  Table 1 lists the distribution of documents, sentences, and drugs as contained in the training and test set of DDI2011 [6]. Since there is only one type of entity names (DRUG) in this corpus, the text would be only labeled as “B/I-DRUG” or “O”.

For further performance evaluation of the proposed model, the SemEval-2013 dataset in drug name recognition and classification task was used.  Table 2 shows the numbers assigned to the annotated entities in DDI2013 training set and test set. The dataset contains four entity types: Drug, Brand, Group, and Drug_n [43]. Drug denotes any chemical reagent served to treat, cure, prevent or diagnose human diseases. Brand is characterized by trade name or brand name. Group denotes any term that specifies the chemical or pharmacological relations between a group of drugs as mentioned in the text, and Drug_n describes a kind of chemical reagent that has not been approved for human medical use.

### 4.2. Pretrained Embedding

In this work, Pennington et al. [25] was used to initialize the word embedding obtained from the pretraining on PMC and PubMed, and the context-sensitive word vectors were acquired using ELMo. The character embedding was randomly initialized according to a uniform sample $\left[-\sqrt{\left(3/\text{dim}\right)},+\sqrt{\left(3/\text{dim}\right)}\right]$, where dim = 30.

### 4.3. Hyperparameters

Table 3 lists the hyperparameters used in the course of experiment. The dimensions of pretrained word embedding, character embedding, and contextualized character embedding were set to 30, 100, and 1024, respectively. In the training process, the parameters were updated using Minibatch Stochastic Gradient Descent (SGD) in respect of descending learning rate. The initial learning rates of the proposed model, Dropout rate, and the batch size were set to 0.015, 0.5, and 10, respectively.

### 4.4. Criteria for Evaluation

In the experiment, the system performance was evaluated by precision, recall rate, and *F*1. Precision represents all correctly predicted entities as a percentage of all predicted entities. Recall rate represents the predicted entities as a percentage of all entities as contained in the dataset. *F*1 represents the harmonized mean value of precision and recall rate, with the following equation:

(7) $$\begin{array}{c} P=\frac{\text{TP}}{\text{TP}+\text{FP}},\\ R=\frac{\text{TP}}{\text{TP}+\text{FN}},\\ F1=\frac{2*P*R}{P+R}, \end{array}$$

where TP denotes the number of true-positive samples, TN denotes the number of true-negative samples, FP denotes the number of false-positive samples, and *F* denotes the number of false-negative samples. Two out of four criteria for evaluation available in DDI2013 [43] Challenge Corpus were used: type matching (only if there are some overlaps with the same category of gold drug names) and strict matching (only if the label boundary and category are the same as the gold drug names, the label drug names are correct).

## 5. Experiment and Analysis

The multi-DTR model as described here was evaluated on DDI2011 and DDI2013, known as the representative biomedical corpora.  Table 4 is the performance comparison of multi-DTR with the works done by other teams. Next, the impact of each architecture (e.g., different embedded layers, different optimization methods, and multitask mutual feedback framework) as a part of the proposed model on the experiment was assessed. The findings of comparison suggest that the architectures of the proposed model would perform well in the experiment.

### 5.1. Performance Comparison with Available Methods

The results were compared with those of the works done by other teams. For the sake of fairness and rationality of the experiment, the hyperparameters of the proposed model were configured according to the optimal parameters as referred to in the article. As is seen from Table 4, the dictionary-based method and the rule-based method, as proposed earlier, yielded reasonable results, including Tsuruoka [12] and Hettne et al. [13], subsequent deep learning model. For example, LASIGE et al. [43] combined CRF with the list of dictionary terms intended for DNER processing as collected from the database in order to recognize and classify entities. Zeng et al. [16]used the BiLSTM-CRF structure to identify drug entities without the aid of any external dictionary, with good results attained. Yang et al. [37] used a hierarchical recursive network for cross-language transfer learning. The model proposed by Liu et al. [44] combines the word embedding trained in biomedical text with the semantic features of three drug dictionaries, with an impressive performance on DDI2013, suggesting that the accuracy of our proposed model is 0.90% lower than that proposed by Liu et al. [44], but its recall rate and *F*1 are 6.23% and 2.43% higher than that proposed by Liu [44].

For the evaluation of DDI2013 dataset, Table 5 provides a summary of the accurate evaluation of the proposed model in the entity type-specific recognition as part of DDI2013.

Despite good performance in type recognition, the proposed model may neglect the difference between a given entity and other entity types due to a small percentage (<4%) of Drug_n entity type in the dataset. As a result, the recognition accuracy of the proposed model would be lower than that of any other entity.

### 5.2. Performance Comparison of Different Statements

This work proposed using pretrained word embedding, character representation, and context-sensitive word embedding to obtain additional feature information, as given in Table 6. To test the impact of different input information representations on the proposed model, three kinds of embedding information were combined and input into the model, respectively. According to the results, serial representation is better than single representation, and multiple representations can attain the best performance.

### 5.3. Comparison of Optimization Methods

Different optimizers, including SGD, AdaGrad, Adadelta, RMSProp, and Adam, were compared here. SGD can calculate gradient and update parameters by randomly extracting the training sample of a fixed size while avoiding falling into saddle points or poor local optimal points. AdaGrad imposes a constraint on the optimal learning rate and is suitable for processing sparse gradient, but it may cause the disappearance of gradient. Adadelta is an extension of AdaGrad and simplifies the computational process. RMSProp relies on a global learning rate and is suitable for processing nonstationary targets. Adam can adjust the parameter-specific learning rate using first-order moment estimation and second-order moment estimation, but it is vulnerable to generalization and convergence problems. According to the experimental results, as given in Figure 5, SGD is significantly better than any other optimizer.

### 5.4. Performance Comparison in Case of Dropout

The effectiveness of Dropout was evaluated here, with all of the other hyperparameters in the model identical to that in Table 3. As given in Table 7, the performance of the proposed model on DDI2011 and DDI2013 was slightly improved after the Dropout was used, which in turn proves that Dropout plays a part in reducing overfitting.

### 5.5. Performance Comparison between Multitask Learning and Single-Task Learning

The effectiveness of multitask learning strategy was also examined. As seen from Table 8, the efforts to jointly model DNER and DNEN by using two explicit feedback strategies would significantly improve the model performance, partly because the multitask learning provides a general representation of both tasks and partly because the proposed method converts hierarchical tasks into parallel multitask setting and retains mutual support between different tasks.

## 6. Conclusion

Drug text mining is a key interdisciplinary field of computer science and biomedicine. In this work, a multitask learning framework was tailored for DNER, with an impressive performance on DDI2011 and DDI2013. Through detailed analysis, the main gains of the proposed model can be attributed to character sharing between drug entities, pretrained word embedding, and context-sensitive word embedding information. The conflict of entity boundary and type can be generally resolved by the positive feedback of DNER and DNEN. According to the experimental results, the proposed method can readily perform well without the aid of any drug dictionary or manual creation so an efficient DNER system was constructed.

## Figures and Tables

**Figure 1:** An example of DNER and DNEN tasks.

**Figure 2:** CNN used to extract a character-level representation of words.

**Figure 3:** Structure of the ELMo model.

**Figure 4:** The main architecture of the multi-DTR model.

**Figure 5:** Performance comparison of different optimization methods optimization.

**Table 1:** Training and testing set in DDI2011.

Set	Documents	Sentences	Drugs
Training	435	4267	11260
Final test	144	1539	3689
Total	579	5806	14949

**Table 2:** Numbers of the annotated entities in DDI2013 set.

Type	Train			Test		
	DrugBank	MedLine	Total	DrugBank	MedLine	Total
Drug	9901 (63%)	1745 (63%)	11646 (63%)	180 (59%)	171 (44%)	351 (51%)
Brand	1824 (12%)	42 (1.5%)	1866 (10%)	53 (18%)	6 (2%)	59 (8%)
Group	3901 (25%)	324 (12%)	4225 (23%)	65 (21%)	90 (24%)	155 (23%)
Drug_n	130 (1%)	635 (23%)	765 (4%)	6 (2%)	115 (30%)	121 (18%)
Total	15756	2746	18502	304	382	686

**Table 3:** The parameters for our experiments.

Layer	Hyperparameter	Value
CNN	Window size	3
	Number of filters	30

LSTM	State size	200
	Initial state	0.0
	Peepholes	No

Dropout	Dropout rate	0.5
	Batch size	10
	Initial learning rate	0.015
	Gradient clipping	5.0
	Decay rate	0.05
	Labeling schema	BIO
	ELMo dim	1024

**Table 4:** Results of experiment in DDI2011 and DDI2013.

System	DDI2011			DDI2013		
	Precision	Recall	*F*1	Precision	Recall	*F*1
UMCC_DLS	－	－	－	24.00	57.00	34.00
Hettne	66.91	71.42	69.09	59.41	56.32	57.82
Tsuruoka	68.42	72.39	70.34	62.24	58.17	60.12
WBI	89.53	88.42	88.97	76.70	88.42	74.80
LASIGE	87.02	82.51	84.70	78.00	56.00	65.19
Yang	81.44	81.50	81.46	76.54	74.40	75.45
Zeng	93.26	91.11	92.17	83.60	77.81	79.26
Liu	－	－	－	87.46	75.22	80.88
Multi-DTR	94.36	92.13	93.22	85.56	81.45	83.45

**Table 5:** Experimental results of different entity types in DDI2013.

Type	Precision	Recall	*F*1
Drug	86.52	81.68	84.03
Brand	89.46	78.51	83.62
Group	83.26	86.43	84.81
Drug_n	79.74	67.36	73.02
Mico-average	85.56	81.45	83.45

**Table 6:** Performance comparison of each representations.

System	DDI2011			DDI2013		
	Precision	Recall	F1	Precision	Recall	F1
ELMo	88.46	87.74	88.09	82.14	79.24	81.68
Char	86.32	85.12	85.71	81.21	78.53	79.84
Glove	88.12	89.34	88.72	84.74	80.57	82.60
ELMo + Char	89.47	90.55	90.00	83.45	81.06	82.23
Char + Glove	90.14	88.42	89.24	83.32	80.64	81.95
ELMo + Glove	91.73	89.51	90.60	84.24	81.32	82.75
ELMo + Glove + Char	94.36	92.13	93.22	85.56	81.45	83.45

**Table 7:** Performance comparison using Dropout.

		Precision	Recall	F1
DDI2011	No	92.73	91.11	91.91
	Yes	94.36	92.13	93.22
	Δ	+1.63	+1.02	+1.31

DDI2013	No	83.52	79.71	81.04
	Yes	85.56	81.45	83.45
	Δ	+2.04	+1.74	+2.41

**Table 8:** Performance comparison of adopting multitask learning.

		Precision	Recall	*F*1
DDI2011	Single-task	91.13	89.51	90.30
	Multitask	94.36	92.13	93.22
	Δ	+3.23	+2.62	+2.92

DDI2013	Single-task	83.42	78.01	80.62
	Multitask	85.56	81.45	83.45
	Δ	+2.14	+3.44	+2.83

## Data Availability

The experimental datasets used in this work are publicly available, and the bundled data and code of this work are available from the corresponding author upon request.
